The article "Altering the inhibitory kinetics and molecular conformation of maltase by Tangzhiqing (TZQ), a natural α-glucosidase inhibitor" was published in 2020. Journal: BMC Complement Med Ther.

# Altering the inhibitory kinetics and molecular conformation of maltase by Tangzhiqing (TZQ), a natural α-glucosidase inhibitor

**DOI:** 10.1186/s12906-020-03156-3

**Published:** 2020-11-18

**Authors:** Yanfen Li, Xiaomao Zhang, Ruihua Wang, Lu Han, Wei Huang, Hong Shi, Baohe Wang, Ziqiang Li, Shaolan Zou

**Affiliations:** 1 Second Affiliated Hospital of Tianjin University of Traditional Chinese Medicine, No.69 Zengchan Road, Hebei District, Tianjin, 300250 China; 2 School of Chemical Engineering and Technology, Tianjin University, No. 135 Yaguan Road, Jinnan District, Tianjin, 300350 China; 3 Tianjin University of Traditional Chinese Medicine, No. 10 Poyanghu Road, Tuanbo New Town, Jinghai District, Tianjin, 301617 China

## Abstract

**Background:**

Tangzhiqing (TZQ), as a potential α-glycosidase inhibitor, possesses postprandial hypoglycaemic effects on maltose in humans. The aim of this study was to investigate the mechanisms by which TZQ attenuates postprandial glucose by interrupting the activity of maltase, including inhibitory kinetics and circular dichroism studies.

**Methods:**

In this study, we determined the inhibitory effect of TZQ on maltase by kinetic analysis to determine the IC_50_ value and enzyme velocity studies and line weaver-burk plot generation to determine inhibition type. Acarbose was chosen as a standard control drug. After the interaction with TZQ and maltase, secondary structure analysis was conducted with a circular dichroism method.

**Results:**

TZQ showed notable inhibition activity on maltase in a reversible and competitive manner with an IC_50_ value of 1.67 ± 0.09 μg/ml, which was weaker than that of acarbose (IC_50_ = 0.29 ± 0.01 μg/ml). The circular dichroism spectrum demonstrated that the binding of TZQ to maltase changed the conformation of maltase and varied with the concentration of TZQ in terms of the disappearance of β-sheets and an increase in the α-helix content of the enzyme, similar to acarbose.

**Conclusions:**

This work provides useful information for the inhibitory effect of TZQ on maltase. TZQ has the potential to be an α-glycosidase inhibitor for the prevention and treatment of prediabetes or mild diabetes mellitus.

## Background

Elevated postprandial glucose, which is one of the earliest abnormalities of glucose homeostasis associated with diabetes, will increase the risk of developing microvascular complications and cardiovascular disease [1, 2]. Postprandial glycaemia often accompanies several long-term complications, such as nephropathy, hypertension, atherosclerosis and hyperlipidaemia [3]. Diabetes mellitus is becoming a serious threat to human health worldwide [4]. One encouraging approach for better control of postprandial glycaemia is to reduce carbohydrate digestion [5]. The clinically used α-glucosidase inhibitors, including acarbose, miglitol and voglibose, can bind to α-glucosidase and competitively inhibit the enzyme in the small intestine to delay the expeditious generation of blood glucose [1, 6].

As a Chinese herbal medicine, Tangzhiqing (TZQ) is composed of *Nelumbonucifera* Gaertn. leaves, *Paeonialactiflora* Pall. roots, *Salviamiltiorrhizabge.* roots, *Morus alba* L. leaves, and *Crataeguspinnatifidabge.* leaves and has a long history of use in treating diabetes mellitus. Based on the recipe of TZQ, we developed a new formula including eight fractions of red paeony saponins, lotus leaf alkaloids, lotus leaf flavonoids, mulberry leaf alkaloids, mulberry leaf flavonoids, mulberry leaf polysaccharide, danshen polyphenols, and hawthorn leaf flavonoids with a ratio of 3.0:2.9:1.8:0.8:0.1:14.0:0.8:0.2 (w/w) [7]. The fractions of mulberry leaf alkaloids, mulberry leaf flavonoids, and hawthorn leaf flavonoids significantly inhibited glucose absorption. The TZQ formula possesses the effects of anti-hyperlipidaemia, anti-hyperglycaemia, and anti-oxidative stress, which suggests that TZQ could be developed as a potential ready-made formula for pre-diabetes treatment [7–9]. Moreover, the TZQ formula was used in an Investigational New Drug Application study by the China Food and Drug Administration in November 2010.

Preclinical studies have shown that TZQ has obvious inhibitory effects on rat intestinal saccharase for sucrase and maltase in vivo [8]. In genetically modified KK-Ay mice with type 2 diabetes, TZQ presented beneficial effects on the improvement of glucose metabolism by reducing α-glycosidase activity [9]. TZQ has the same effects as acarbose, which inhibits the postprandial increase in blood glucose levels by inhibiting and delaying digestion and absorption of carbohydrates in healthy Chinese volunteers. Moreover, TZQ was found to significantly regulate abnormal glucose, decrease insulin secretion to maintain normoglycaemia, and reduce glycosylated haemoglobin (HbA1c) and fasting insulin in type 2 diabetes mellitus patients [10, 11]. An eight-period, self-crossover clinical trial in healthy volunteers was performed to determine the effect of TZQ on the glycaemic index (GI) of common carbohydrates. The results proved that TZQ could decrease the GI of sucrose, maltose and starch. For maltose, 6 tablets of TZQ were the best dose, and the activity of maltase was inhibited. Based on these results, this study aimed to investigate the mechanisms of TZQ action on maltase by measuring maltase inhibitory activity, conducting kinetics assays and determining the secondary structures of maltase via circular dichroism (CD). Acarbose was used as a control drug. This study will provide a scientific basis for TZQ treatment of diabetes and useful in new drug development.

## Methods

### Materials

Maltase (EC: 3.2.1.20) was purchased from Shanghai Yuanye Bio-Technology Co., Ltd. (Shanghai China). Acarbose was obtained from the National Institutes for Food and Drug Control (Beijing, China). Maltose was purchased from TS Corporation (Seoul, Korea). TZQ extract was provided by Shandong Buchang Shenzhou Pharmaceutical Co., Ltd. The content of TZQ was determined by the chemical marker component of hypericin (10 mg/g TZQ). All other reagents and solvents were of analytical reagent grade, and ultrapure water was used throughout the experiment.

### Excess concentration of the substrate, optimum concentration of the enzyme and optimum reaction time

Ten microlitres of maltase (5 mg/mL) was reacted with maltase substrates at different concentrations (0.0125, 0.025, 0.05, 0.1, 0.175, 0.25, 0.40, and 0.55 mol/L) at 37 °C for 10 min and cooled for 5 min. Sodium carbonate buffer was added to stop the reaction according to the operation steps of the glucose assay kit. The absorbance was measured at 492 nm. Excess maltose was used in the following study. A total of 90 μL of 0.25 mol/L maltose solution was added to 10 μL of different concentrations of maltase (0.3125, 0.625, 1.25, 2.5, 5, 10, and 20 mg/ml) at 37 °C, and sodium carbonate was added to stop the reaction from 2 min to 16 min in 2 min intervals. The absorbance was measured at 492 nm with an INFINITE F50 Enzyme standard instrument (TECAN, Switzerland).

### Maltase inhibition assay

A 15 μL sample solution at various concentrations (6.25 × 10^− 4^, 1.25 × 10^− 3^, 2.5 × 10^− 3^, 5 × 10^− 3^, 1 × 10^− 2^, 2 × 10^− 2^, 4 × 10^− 2^, and 5 × 10^− 2^ mg/mL) in ultrapure water was premixed with 10 μL of maltase solution (5 mg/ml) dissolved in sodium phosphate buffer (Ph = 6.0) and incubated at 37 °C for 10 min. Then, 75 μL of preheated maltose solution was added to start the reaction. The reaction was carried out at 37 °C for 12 min and terminated by the addition of 100 μL of sodium carbonate [12]. The mixture was cooled for 5 min. After cooling and centrifugation at 10000 rpm for 10 min, a chromogenic agent was added to the supernatant, and the absorbance was measured at 492 nm. Acarbose was used as a positive control drug for this assay at concentrations of 5 × 10^− 4^, 1 × 10^− 3^, 2 × 10^− 3^, 2.2 × 10^− 3^, 2.4 × 10^− 3^, 2.6 × 10^− 3^, 4 × 10^− 3^, and 5 × 10^− 3^ mg/ml.

The enzymatic activity assayed without TZQ or acarbose was defined as 100% relative activity. Relative enzymatic activity (%) = (slope of reaction kinetics equation obtained by reaction with TZQ or acarbose)/(slope of reaction kinetics equation obtained by reaction without TZQ or acarbose)*100% [13, 14]. The percent inhibition [%] was obtained using the following equation:

$$ \mathrm{Inhibition}=\left(\mathrm{Ac}-\mathrm{As}\right)/\mathrm{Ac}\ast 100\% $$

where Ac is the absorbance of the control and As is the absorbance of the sample [15]. The inhibition was plotted against the sample concentration, and the half inhibitory concentration (IC_50_) value was calculated from the regression curve. The IC_50_ of TZQ or acarbose was the concentration of TZQ or acarbose causing a loss of 50% of the enzyme activity. The IC_50_ value was calculated from three independent assays performed in triplicate.

### Inhibitory kinetic analysis

The reaction mixtures (100 μL) containing 15 μL of TZQ (C = 0.032 mg/ml) and 2–16 μL of maltase solution (5 mg/mL) were preincubated for 10 min at 37 °C, and the reaction was started by the addition of 65 μL of maltose. Then, 100 μL of sodium carbonate solution was added to stop the reaction 12 min after cooling for 5 min. Absorbance was measured later. The initial velocity (*V*) for a set volume of enzyme (E) was determined. Acarbose (15 μL, 0.002 mg/mL) was used as a positive control drug, and sodium phosphate buffer (15 μL, pH = 6.0) was used as a negative control.

To further explore the inhibitory characteristics of TZQ, enzyme kinetic analysis was performed according to the above reaction using Line weaver-Burk plots of 1/V versus 1/[S]. The quantity of maltase was maintained at 10 μL (5 mg/mL), and 15 μL of sample (0.020, 0.030 mg/ml) was measured in various concentrations of maltose (0.025–0.2 mol/L). Km and Vmax were obtained from double-reciprocal line-weaver burk plots [16]. Acarbose (10 μL, 0.002 mg/mL) and sodium phosphate buffer (15 μL, pH = 6.0) were used as positive and negative controls, respectively.

### Circular dichroism measurement

Circular dichroism (CD) experiments were carried out at a constant temperature of 25 °C with a Jasco J-810 spectropolarimeter equipped with a Model PTC-423S/L Peltier type temperature controller. A 0.1 cm path-length cuvette was used. Each sample was scanned at least three times to obtain the average within the wavelength range of 190–250 nm, and points were taken in 1 nm intervals. The enzyme solution was prepared at a concentration of 1.0 mg/mL in 20 mM potassium phosphate buffer (pH = 7). TZQ concentrations were between 0.07 and 0.28 g/L, and acarbose was used at 0.5 g/L. CD spectra were measured at different time intervals after the addition of TZQ or acarbose into the enzyme solution. The secondary structures of maltase, including α-helices, β-sheets, β-turns and random coils, were analysed by the Chen-Yang program.

### Statistical analysis

All analyses were performed on the original dates, which were repeated at least three times, and the results are expressed as the mean ± SD. All data were analysed with Student’s t-test using GraphPad Prism version 6.0 for Windows (GraphPad Software, San Diego California, USA). Typical spectra and data are presented as figures.

## Results

### Selection for concentration of the substrate, optimum enzyme concentration and action time

The reactions were implemented at 37 °C and sodium phosphate buffer was maintained at pH 6.0. When the substrate (maltose) concentration remained at a low level (< 0.1 mol/L), as shown in Fig. 1, the reaction rate was directly proportional to the substrate concentration, indicating a first-order reaction. The mixed-order reaction was observed when the concentration was between 0.1 mol/L and 0.175 mol/L, and the zero-order reaction was maintained for the proper substrate concentration (> 0.175 mol/L), so the excess concentration of the substrate was 0.25 mol/L. The linear reaction time of maltase decreased gradually with increasing maltase concentration (Fig. 2). When the concentration of maltase was 5 mg/mL or below, the reaction was linear within 12 min. The initial rate of the reaction was further compared, and the kinetics of the enzyme reaction were analysed by the optimal maltase concentration (5 mg/mL) and the reaction time (12 min).

**Fig. 1:** Effect of maltose at different concentrations on the reaction rate of maltase at a wavelength of 492 nm

**Fig. 2:** Curves of reaction progress of maltase vs. time at different concentrations

### Comparison of TZQ and acarbose on maltase activity

The activity of maltase was significantly inhibited by various concentrations of TZQ in a concentration-dependent manner (Fig. 3a). As the positive control drug, the influence of acarbose is shown in Fig. 3b. The concentrations of TZQ and acarbose resulting in 50% maltase activity loss (IC_50_) were estimated to be 1.67 ± 0.09 and 0.29 ± 0.01 μg/ml, respectively (*P* < 0.05, by logistic regression curve). The results suggested that TZQ had weaker maltase inhibitory activity than that of acarbose.

**Fig. 3:** Inhibitive curves of TZQ (**a**) and acarbose (**b**) on maltase

### Inhibition mechanism

If the inhibition is reversible, the plots of *V* versus enzyme concentration would pass through the origin [17]. The plots of *V* vs. maltase at different concentrations of TZQ and acarbose are shown in Fig. 4. It was shown that all the straight lines passed through the origin of the coordinate axis, including those of the TZQ, negative control (sodium phosphate buffer) and positive control (acarbose) samples. The plots indicated that the inhibition of maltase by TZQ was reversible, similar to that of acarbose.

**Fig. 4:** Kinetic curves of inhibition of maltase by TZQ (**a**) and acarbose (**b**)

To further investigate the inhibitory mechanism of TZQ, Dixon plots in which the reciprocal of the rate of the reaction was plotted against the inhibitor concentrations were generated (Fig. 5a). It was shown that TZQ exhibited a competitive inhibition mechanism on maltase as the lines for substrate concentrations converged near the *y*-axis [18], the *V*_max_ value remained 0.30 mmol/L·min, and the *K*_m_ value changed from 0.19 to 0.22 mol/L, which were computed from the double-reciprocal Line weaver-Burk plot. This behaviour was similar to that of acarbose (Fig. 5b), which also showed a competitive inhibition mechanism.

**Fig. 5:** Line weaver-Burk plots of reversible inhibition of TZQ (**a**) and acarbose (**b**) on maltase

### Circular dichroism measurements

To clarify the pathway and mechanism behind the effect of TZQ on human bodies, CD spectra of maltase with/without TZQ were collected, including far-UV between 190 and 250 nm. The optional dose of TZQ was 0.07 ~ 0.28 g/L. TZQ was proven to be suitable for the CD assay in our preliminary study. The results are shown in Fig. 6a-c, and the contents of secondary structures are shown in Table 1. These data clearly indicated a similar change between different TZQ concentrations and processing times. While the CD density slightly changed with the addition of TZQ, the peak position and shape significantly varied with time, especially for 0.14 g/L TZQ (Fig. 6b). As a result, the α-helix content of the enzyme increased, with a maximum of 47.9%, and the β-sheet content decreased accordingly and was even undetectable (Table 1). At the same time, while the random structure remained almost constant, the proportion of β-turns also decreased. After the addition of TZQ into the enzyme solution, single CD scanning under the aforementioned conditions was performed for 5 min. The difference before and after addition was undoubtedly obvious, implying that TZQ could rapidly act on maltase and influence activity by conformational changes. As a positive control, the results for acarbose binding are shown in Fig. 6d and Table 2.

**Fig. 6:** Secondary structure of maltase with or without 0.07, 0.14, and 0.28 g/L TZQ are presented in figures **a**, **b**, and **c**, respectively, as well as the positive control acarbose (0.5 g/L, **d**)

**Table 1:** Secondary structure of maltase with and without 0.07, 0.14, and 0.28 g/L of TZQ at different times

Secondary structure	0 min	5 min			45 min		
	without TZQ	TZQ (0.07 g/L)	TZQ (0.14 g/L)	TZQ (0.28 g/L)	TZQ (0.07 g/L)	TZQ (0.14 g/L)	TZQ (0.28 g/L)
α-helix(%)	27.90	31.30	39.60	32.50	38.90	40.80	47.90
β-sheet(%)	25.10	14.80	10.60	7.20	0.00	5.10	0.00
β-turn(%)	9.20	20.60	16.40	23.30	24.20	20.80	17.40
Random coil(%)	37.80	33.30	33.40	36.90	36.90	33.30	34.70
Total(%)	100.00	100.00	100.00	100.00	100.00	100.00	100.00

**Table 2:** Secondary structure of maltase with and without acarbose (0.5 g/L) at different time

Secondary structure	0 min	5 min	45 min
α-helix(%)	27.90	34.60	34.40
β-sheet(%)	25.10	19.60	4.40
β-turn(%)	9.20	10.00	22.00
Random coil(%)	37.80	35.80	39.20
Total (%)	100.00	100.00	100.00

## Discussion

The delayed absorption of glucose is one of the principal therapeutic approaches for type 2 diabetes. The α-glucosidase inhibitors compete with the α-glucosidase enzyme activity, which helps to reduce the conversion of carbohydrates into glucose and thereby control postprandial hyperglycaemia incidence [19, 20]. Currently prescribed α-glucosidase inhibitors, such as acarbose, voglibose, and miglitol, have depicted different side effects, including bloating, diarrhoea, flatulence, pain, and abdominal discomfort [21].

This study qualitatively and quantitatively investigated the mechanism of hypoglycaemia by TZQ, a Chinese herbal medicine, for the first time. We utilized maltase as a target, and in vivo data provided evidence of the effect of TZQ on the reduction in postprandial glycaemia following maltose consumption. IC_50_ values and kinetic parameters from Line weaver-Burk double-reciprocal-plots and Dixon plots were used as approaches to enzyme inhibition [22]. The results showed that TZQ exhibited an obvious inhibition against maltase, similar to acarbose, flavonoids in the leaves of *Morus atropurpurea* and 1-deoxynojirimycin (DNJ) [23, 24]. DNJ and flavonoids in mulberry leaves were reported to be alkaloid and flavone components in TZQ, and the results for rats were similar to those observed in this study [7]. However, TZQ had no side effects of abdomen expansion and exhaust compared with acarbose [10].

When invertibility persisted, a straight line through the origin was obtained because the quantity of inhibitors was constant. If the inhibition was irreversible, the enzyme was inactivated by covalent binding between the inhibitor and enzyme and formed a stable complex. Thus, the plots of *V* versus enzyme concentration would not pass through the origin [17]. This study proved that the inhibition of maltase by TZQ was reversible, similar to acarbose. For competitive inhibition, the lines for substrate concentrations would converge at the y-axis or x-axis when competitive inhibition or non-competitive inhibition existed [18]. For anticompetitive inhibition, the lines are parallel. When a mixed inhibition mechanism existed, the data lines intersect in the second or third quadrant on the Line-weaver Burk plots [24–26]. The results showed that the substrate concentration lines intersected at the y-axis, and with the increase in the concentration of TZQ, no change was observed in the *V*_max_ values, while the *K*_m_ values increased, indicating that this sample acted as a competitive inhibitor, similar to acarbose [27–29]. Our previous studies showed that the fractions mulberry leaf alkaloids, mulberry leaf flavonoids, and hawthorn leaf flavonoids show strong inhibitory effects on rat intestinal maltase [7]. In particular, the fraction of mulberry leaf alkaloids (IC_50_ = 0.05 μg/ml for maltase) is stronger than that of the positive control acarbose (IC_50_ = 0.75 μg/ml) [7]. The extract from leaves of *Morus alba* displayed competitive maltase inhibition [30]. Salvianolic acid A reversibly inhibited maltase in a competitive manner, and the inhibition exhibited a multiphase kinetics process with a first-order reaction [31]. Additionally, the inhibitory constant of the DNJ equivalent for maltase was 2.1 × 10^− 4^ mM, and the inhibitory activity was shown to be competitive [32]. However, Wu et al. reported that DNJ reversibly inhibited the activity of maltase in a mixed-type manner with an IC_50_ of (1.5 ± 0.1) μM and an inhibition constant Ki of (2.01 ± 0.02) μM [24]. Competitive inhibition behaviour has been reported for some active fractions and ingredients in previous studies [32], which is the same result as the TZQ sample used in the current study. Therefore, it was concluded that the inhibition of maltase by TZQ was competitive. For competitive inhibition, the inhibitor competes for the active site of an enzyme with the substrate, different from other types of inhibition [33, 34]. In mixed and non-competitive inhibition mechanisms, the inhibitor binds to both the free enzyme and enzyme-substrate complex. However, non-competitive inhibitors present the same affinity towards enzyme and enzyme-substrate complexes, while mixed-type inhibitors have different affinities for these two constituents [35]. This behaviour was the same as that of acarbose, which was reported by Hao He and Yan-Hua [1].

CD spectroscopy is a sensitive technique to monitor the conformational changes in proteins upon interaction with a ligand [36]. The results indicated that the binding of TZQ to maltase resulted in molecular conformational changes in maltase, which led to the inactivation of maltase (Fig. 6a-c). Interestingly, the effect of DNJ on the contents of α-helix and β-sheet secondary structures in maltase was reported to be different by Hao Wu et al. [24] and by Hao He and Yan-Hua Lu [1]. Our results were similar to those from the latter group. DNJ, an abbreviation for 1-deoxynojirimycin, was reported to be a main alkaloid component in TZQ [7] and could inhibit maltase activity [1, 24]. It is well known that acarbose is often used as a positive control in drug tests. Here, acarbose was also selected as a control to investigate its effect on maltase. The results demonstrated a similar tendency for both TZQ and acarbose to decrease the β-sheets and increase the α-helix content of the enzyme. These results proved the similar mechanism of TZQ and acarbose on the inhibition of maltase.

Unravelling the conformational changes in enzymes together with inhibition kinetics during an enzymatic reaction has great potential in researching therapeutic drugs [37]. The present study provided evidence to understand the basis of TZQ as an α-glycosidase inhibitor, its inhibition mechanism and that the inhibition activities are reversible and competitive. Our results suggested that TZQ is useful to protect against hyperglycaemia by inhibiting the activity of maltase. However, it is unclear which ingredients in TZQ are responsible for the α-glycosidase inhibitor activity. In previous studies, we tentatively characterized 46 ingredients from the TZQ formula [38]. Additionally, nuciferine and paeoniflorin have been identified as promising Q-markers/PK-markers of TZQ based on fingerprint qualitative analysis, multicomponent quantitative analysis, and dose-exposure-response analysis [38, 39]. Therefore, we plan to conduct the same investigation on the Q-markers/PK-markers of TZQ to identify which ingredients are responsible for α-glycosidase inhibitor activity.

## Conclusions

This paper proved that TZQ exhibited an invertibility and competitive inhibition mechanism on maltase. The characteristics were similar to those of acarbose. Molecular conformations in the CD spectra showed that their binding resulted in conformational changes of maltase, characterized by an increase in α-helix structures and a decrease in β-sheet structures, which was similarly observed for acarbose. Our study provides a basis for the application of TZQ as a natural plant product to treat prediabetes or mild diabetes mellitus as an α-glycosidase inhibitor.

## Data Availability

The data used to support the findings of this study are available from the corresponding author upon reasonable request.

## Abbreviations

TZQ: Tangzhiqing
GI: Glycaemic index
IC_50_: Half inhibitory concentration
CD: Circular dichroism

## References

[1] He H, Lu Y-H (2013). Comparison of inhibitory activities and mechanisms of FiveMulberry plant bioactive components against α-Glucosidase. Agric Food Chem.

[2] Danaei G, Finucane MM, Lu Y, Singh GM, Cowan MJ, Paciorek CJ (2011). National, regional, and global trends in fasting plasma glucose and diabetes prevalence since 1980: systematic analysis of health examination surveys and epidemiological studies with 370 country-years and 2.7 million participants. Lancet.

[3] Goh SY, Cooper ME (2008). Clinical review: the role of advanced glycation end products in progression and complications of diabetes. J Clin Endocrinol Metab.

[4] Chen L, Magliano DJ, Zimmet PZ (2011). The worldwide epidemiology of type 2 diabetes mellitus–present and future perspectives. Nat Rev Endocrino.

[5] Beejmohun V, Peytavy-Izard M, Mignon C, Muscente-Paque D, Deplanque X, Ripoll C (2014). Acute effect of Ceylon cinnamon extract on postprandial glycemia: alpha-amylase inhibition, starch tolerance test in rats, and randomized crossover clinical trial in healthy volunteers. BMC Complement Altern Med.

[6] Worawalai W, Sompornpisut P, Wacharasindhu S, Phuwapraisirisan P (2016). Voglibose-inspired synthesis of new potent α-glucosidase inhibitors N-1,3-dihydroxy propylaminocyclitols. Carbohydr Res.

[7] Tao W, Deqin Z, Yuhong L, Hong L, Zhanbiao L, Chunfeng Z (2010). Regulation effects on abnormal glucose and lipid metabolism of TZQ-F, a new kind of traditional Chinese medicine. J Ethnopharmacol.

[8] Wang T, An YT, Zhao CF (2011). Regulation effects of crataegus pinnatifida leaf on glucose and lipids metabolism. J Agric Food Chem.

[9] Wang W, Miura T, Shi H, Ma DM, Zhao QD, Zhang WP (2008). Effect of Tangzhiqing on glucose and lipid metabolism in genetically type 2 diabetes KK-ay mice. J Health Sci.

[10] Yuhong H, Wenxu F, Yanfen L, Yu L, Ziqiang L, Liu Y (2014). Comparison of the effects of Acarbose and TZQ-F, a new kind of traditional Chinese medicine to treat diabetes, Chinese healthy volunteers. Evid-Based Compl Alt Med.

[11] Liu J, Li Z, Liu H, Wang X, Lv C, Wang R (2018). Metabolomics-based clinical efficacy and effect on the endogenous metabolites of Tangzhiqing tablet, a Chinese patent medicine for type 2 diabetes mellitus with hypertriglyceridemia. Evid-Based Compl Alt Med..

[12] Sheng Z, Dai H, Pan S, Wang H, Hu Y, Ma W (2014). Isolation and characterization of an α-Glucosidase inhibitor from Musa spp. (Baxijiao) flowers. Molecules..

[13] Lin L, Dong Y, Zhao H, Wen L, Yang B, Zhao M (2011). Comparative evaluation of rosmarinic acid, methyl rosmarinate and pedalitin isolated from Rabdosia Serra (MAXIM.) HARA as inhibitors of tyrosinase and alpha-glucosidase. Food Chem.

[14] Wang LH, Wang MS, Zeng XA, Gong DM, Huang YB (2017). An in vitro investigation of the inhibitory mechanism of β-galactosidase by cinnamaldehyde alone and in combination with carvacrol and thymol. Biochim Biophys Acta.

[15] Zhang YL, Luo JG, Wan CX, Zhou ZB, Kong LY (2015). Four new flavonoids with a-Glucosidase inhibitory activities from Morus alba var. tatarica. Chem Biodivers.

[16] Gupta S, Mahmood S, Khan RH, Mahmood A (2009). Inhibition of brush border sucrase by polyphenols in mouse intestine. Biosci Rep.

[17] Zeng L, Zhang G, Lin S, Gong D (2016). Inhibitory mechanism of apigenin on α-glucosidase and synergy analysis of flavonoids. J Agric Food Chem.

[18] Wang M, Shi J, Wang L, Hu Y, Ye X, Liu D (2018). Inhibitory kinetics and mechanism of flavonoids from lotus (*Nelumbo nucifera* Gaertn.) leaf against pancreatic α-amylase. Biomac.

[19] Tafesse TB, Moghadam ES, Bule MH, Faramarzi MA, Abdollahi M, Amini M. Study on the interaction of 1,5-diaryl pyrrole derivatives with α-glucosidase; synthesis, molecular docking, and kinetic study. Med Chem. 2019. 10.2174/1573406415666191206100336.10.2174/157340641566619120610033631808390

[20] Joshi SR, Standl E, Tong N, Shah P, Kalra S, Rathod R (2015). Therapeutic potential of α-glucosidase inhibitors in type 2 diabetes mellitus: an evidence-based review. Expert Opin Pharmacother.

[21] Hollander P (1992). Safety profle of acarbose, an α-glucosidase inhibitor. Drugs..

[22] Wang R, Chai WM, Yang Q, Wei MK, Peng Y (2016). 2-(4-Fluorophenyl)-quinazolin-4(3H)-one as a novel tyrosinase inhibitor: synthesis, inhibitory activity, and mechanism. Bioorg Med Chem.

[23] Hong HC, Li SL, Zhang XQ, Ye WC, Zhang QW (2013). Flavonoids with α-glucosidase inhibitory activities and their contents in the leaves of Morus atropurpurea. Chin Med.

[24] Wu H, Zeng W, Chen L, Yu B, Guo Y, Chen G (2018). Integrated multi-spectroscopic and molecular docking techniques to probe the interaction mechanism between maltase and 1-deoxynojirimycin, an α-glucosidase inhibitor. Biol Macromolecules.

[25] Cui Y, Liang G, Hu YH, Shi Y, Cai YX, Gao HJ (2015). Alpha-substituted derivatives of cinnamaldehyde as tyrosinase inhibitors: inhibitory mechanism and molecular analysis. J Agric Food Chem.

[26] Ilyina A, Arredondo-Valdés R, Farkhutdinov S, Segura-Ceniceros EP, Martínez-Hernández JL, Zaynullin R (2014). Effect of betulin-containing extract from birch tree bark on α-amylase activity in vitro and on weight gain of broiler chickens in vivo. Plant Foods Hum Nutr.

[27] Saeedi M, Mohammadi-Khanaposhtani M, Pourrabia P, Razzaghi N, Ghadimi R, Imanparast S (2019). Design and synthesis of novel quinazolinone-1,2,3-triazole hybrids as new anti-diabetic agents: in vitro α-glucosidase inhibition, kinetic, and docking study. Bioorg Chem.

[28] Matsui T, Ueda T, Oki T, Sugita K, Terahara N, Matsumoto K (2001). α-Glucosidase inhibitory action of natural acylated anthocyanins. 1. Survey of natural pigments with potent inhibitory activity. J Agric Food Chem.

[29] Worawalai W, Sompornpisut P, Wacharasindhu S, Phuwapraisirisan P (2016). Voglibose-inspired synthesis of new potent α-glucosidase inhibitors N-1,3- dihydroxypropylaminocyclitols. Carbohydr Res.

[30] Oku T, Yamada M, Nakamura M, Sadamori N, Nakamura S (2006). Inhibitory effects of extractives from leaves of Morus alba on human and rat small intestinal disaccharidase activity. Br J Nutr.

[31] Tang H, Ma F, Zhao D (2019). Integrated multi-spectroscopic and molecular modelling techniques to probe the interaction mechanism between salvianolic acid a and α-glucosidase. Spectrochim Acta A Mol Biomol Spectrosc.

[32] Breitmeier D, Günther S, Heymann H (1997). Acarbose and 1-deoxynojirimycin inhibit maltose and maltooligosaccharide hydrolysis of human small intestinal glucoamylase-maltase in two different substrate-induced modes. Arch Biochem Biophys.

[33] Phan MAT, Wang J, Tang J, Lee YZ, Ng K (2013). Evaluation of α-glucosidase inhibition potential of some flavonoids from Epimedium brevicornum. LWT Food Sci Technol.

[34] Su CH, Lu TM, Lai MN, Ng LT (2013). Inhibitory potential of Grifola frondosa bioactive fractions on α-amylase and α-glucosidase for management of hyperglycemia. Biotechnol Appl Biochem.

[35] Alongi M, Anese M (2018). Effect of coffee roasting on in vitro α-glucosidase activity: inhibition and mechanism of action. Food Res Int.

[36] He Y, Wang XB, Fan BY, Kong LY (2014). Honokiol trimers and dimers via biotransformation catalyzed by Momordica charantia peroxidase: novel and potent a-glucosidase inhibitors. Bioorg Med Chem.

[37] Xu Y, Gao Y, Su Y, Sun L, Xing F, Fan C (2018). Single-molecule studies of allosteric inhibition of individual enzyme on a DNA origami reactor. J Phys Chem Lett.

[38] Li Z, Liu J, Zhang D, Du X, Han L, Lv C, Li Y, Wang R, Wang B, Huang Y (2018). Nuciferine and paeoniflorin can be quality markers of Tangzhiqing tablet, a Chinese traditional patent medicine, based on the qualitative, quantitative and dose-exposure-response analysis. Phytomedicine..

[39] Li Z, Liu J, Li Y, Du X, Li Y, Wang R, Lv C, He X, Wang B, Huang Y, Zhang D (2018). Identify super quality markers from prototype-based pharmacokinetic markers of Tangzhiqing tablet (TZQ) based on in vitro dissolution/ permeation and in vivo absorption correlations. Phytomedicine..

